RETRACTED

# Lung ultrasound score in establishing the timing of intubation in COVID-19 interstitial pneumonia: A preliminary retrospective observational study

**DOI:** 10.1371/journal.pone.0238679

**Published:** 2020-09-03

**Authors:** Xiao Lu, Mao Zhang, Anyu Qian, Luping Tang, Shanxiang Xu

**Affiliations:** 1 Department of Emergency Medicine, Second Affiliated Hospital, Zhejiang University School of Medicine, Hangzhou, China; 2 The Wuhan Critical Care Medical Team from Second Affiliated Hospital, Zhejiang University School of Medicine, Hangzhou, China; Azienda Ospedaliero Universitaria Careggi, ITALY

## Abstract

**Purpose:**

To investigate the role of lung ultrasound score (LUS) in assessing intubation timing for patients with severe acute respiratory syndrome coronavirus 2 (SARS-CoV-2) pneumonia.

**Materials and methods:**

Seventy-two patients with critical coronavirus disease 2019 (COVID-19) were admitted to a makeshift intensive care unit (ICU). All patients underwent bedside lung ultrasonography one to two times per day. The patients were either intubated, treated with noninvasive ventilation (NIV), or given high-flow nasal cannula (HFNC) after a discussion with the multidisciplinary group after their conditions worsened. Bedside lung ultrasound was performed daily after intubation, and patients received mechanical ventilation. Lung ultrasound was performed on days 1, 2, 3, 5, and 7 after patients were admitted to the ICU; if the patient was intubated, LUS determination was performed before intubation within 24 h (T1) and on days 1, 2, 5, and 7 after intubation (T2, T3, T4, and T5, respectively).The goal of this study was to evaluate the severity of lung aeration loss in intubated and non-intubated patients with SARS-CoV-2 pneumonia by ultrasound at different time points within one week.

**Results:**

A total of 16 patients were included in this study, including nine who were intubated and mechanically ventilated and seven patients without intubation. The number of elderly individuals in the intubated group was higher than in the non-intubated group (P < 0.05). In addition, there were more male than female patients in both groups. Patient characteristics (BMI, SOFA, and PaO_2_/FiO_2_ value) were similar between the two groups (P > 0.05). The 28-day mortality rate of intubated patients was higher than that of non-intubated patients; six patients in the intubated group and two patients in the non-intubated group died. Nine intubated patients showed changes in LUS within seven days (n = 9). The mean LUS within 24 h before intubation was 12.8 ± 1.3. LUS was significantly higher on T1 than on T5 (P <0.05), and did not significantly differ from T1 to T4. Comparing LUS between intubated and non-intubated patients on T1 showed that the LUS of intubated patients was significantly higher than that of non-intubated patients (P <0.05). Between the two patient groups, oxygenation index was 140.1 ± 7.7 *vs*. 137.8 ± 5.9 on T1, and the respiratory rate of the two groups was 26 ± 5 *vs*. 28 ± 4 breaths/min. Neither oxygenation index nor RR significantly differed between the two groups.

RETRACTED

**Conclusion:**

LUS may be an effective tool for assessing intubation timing in critically ill patients with Covid-19 interstitial pneumonia.

## Introduction

The coronavirus disease 2019 (COVID-19) outbreak began in December 2019 and rapidly spread to different areas of mainland China. On March 14, 2020, WHO declared COVID-19 a pandemic. The most common and severe complication in patients with COVID-19 is acute hypoxemic respiratory failure or acute respiratory distress syndrome (ARDS), which requires oxygen and ventilation therapies [1]. Some critically ill patients require intubation and invasive ventilation [2]. A number of patients with COVID-19 present with “silent” or “happy hypoxia,” in which the body’s oxygen levels are well below 90%, yet patients are still able to breathe normally. For these patients, there is no shortness of breath, fast or shallow breathing, and likely no signs, symptoms, or sense that something may be wrong. Few studies have addressed the timing of intubation for patients with severe acute respiratory syndrome coronavirus 2 (SARS-CoV-2) pneumonia due to the high mortality of patients treated with invasive ventilation.

The histopathology of initial COVID-19 pneumonia is characterized by alveolar damage, which includes alveolar edema, while the inflammatory component is patchy and mild [3]. The analysis of the available CT data from patients with COVID-19 pneumonia [4] shows largely bilateral lesions, which are patchy and confluent, with a ground glass or mixed consolidative and ground glass pattern. To date, current literature from China and Italy doses not recommend the use of lung ultrasounds to diagnose COVID-19. However, lung ultrasounds are known to potentially assist in monitoring lung conditions [5]. It has also been proven that lung ultrasound findings can be suggestive of a wide range of conditions, including pulmonary edema, pleural effusion, and pneumothorax [6]. Lung ultrasounds have also proven capable of detecting lung lesions before the development of hypoxemia in ARDS patients [7]. Ultrasounds can accurately quantify the loss of pulmonary aeration before, after, and during the weaning trial by calculating the lung ultrasound score (LUS) [8]. One prospective two-center study involving 100 patients has demonstrated that the intensity of lung aeration loss occurring during the weaning trial is predictive of post-extubation respiratory distress within 48 h of extubation. The study found that LUS ≥ 14 could identify patients at high risk of developing post-extubation respiratory distress [9, 10]. Other studies recently found that 80 patients weaned from mechanical ventilation showed a 30% reduction in respiratory distress during post-extubation [11, 12]. However, these studies examined diseases similar to COVID-19, but their findings have not yet been proven in COVID-19.

RETRACTED

This study was designed to retrospectively analyze changes in LUS for 16 critically ill patients with COVID-19. Our study examined COVID-19 patients with interstitial pneumonia, using the clinical application of LUS to assess intubation timing.

## Methods

### Study population and recruitment

A retrospective study was conducted in one makeshift ICU in Wuhan. From February 14, 2020 to March 6, 2020, COVID-19 patients were admitted in the ICU of the Cancer Center of Union Hospital, Tongji Medical College, Huazhong University of Science and Technology. A total of 72 patients with critical COVID-19 who were admitted to this ICU within one month were included in this study. Patients with severe COVID-19 met any of the following criteria: 1. respiratory distress, RR ≥ 30 breaths/min; 2. pulse oxygen saturation (SpO_2_) ≤ 93% on room air in the resting state; 3. arterial partial pressure of oxygen (PaO_2_)/oxygen concentration (FiO_2_) ≤ 300 mmHg (1 mmHg = 0.133 kPa); and 4. > 50% lesion progression within 24 and 48 h on pulmonary imaging. Routine bedside lung ultrasound (one to two times each day) was performed on patients who were treated via non-rebreather mask, non-invasive ventilator, or HFNC after admission to the ICU. The patients were treated according to the guidance for Corona Virus Disease 2019 of China (Editions 6, 7) for antiviral and proprietary Chinese medicine. For patients with acute hypoxemic respiratory failure due to COVID-19, deciding whether to proceed with intubation and invasive ventilation can be challenging. In our ICU, if the patient's condition became more severe during the treatment, the multidisciplinary discussion group (MDT) discussed whether to intubate that patient. After the patients received mechanical ventilation treatment, lung ultrasound assessment was performed daily. Retrospective analysis of LUS of patients at different time points was performed for one week. The patient's gender, age, body mass index (BMI index), sequential organ failure assessment (SOFA score), and 28-day mortality rate were recorded; and the evolution of respiratory parameters between the two groups on time point T1 (lung ultrasound performed before intubation within 24 h) were also recorded. This study was approved by the National Health Commission of China and Ethics Commission of Second Affiliated Hospital, Zhejiang University School of Medicine (KY-2020-186). Written informed consent was waived by the Ethics Commission of the designated hospital for emerging infectious diseases.

RETRACTED

### Lung ultrasound

A Mindray M9 Echography (Mindray Co, ShenZhen, China) and a 2 to 4 MHz round-tipped or convex probe was used for the examination. For each patient, 12 areas in the right and left lung were examined, and as delineated by a parasternal line, anterior axillary line, posterior axillary line, and paravertebral line, the anterosuperior, anteroinferior, laterosuperior, lateroinferior, posterosuperior, and posteroinferior lung regions were identified. Scoring of each area was performed according to the most severe lung ultrasound detected in the corresponding intercostal spaces: 0) normal aeration: presence of lung sliding with horizontal A lines or fewer than two isolated vertical B lines; 1) moderate loss of lung aeration: either multiple well-defined and spaced B1 lines, issued from the pleural line or from small juxtapleural consolidations and corresponding to interstitial edema or coalescent B1 lines or issued from the pleural line or from small juxtapleural consolidations, present in a limited portion of the intercostal space and corresponding to localized alveolar edema; 2) severe loss of lung aeration: multiple coalescent vertical B2 lines issued either from the pleural line or from juxta-pleural consolidations, detected in the whole area of one or several intercostal spaces and corresponding to diffuse alveolar edema; 3) lung consolidation: the presence of a tissue pattern containing either hyperechoic punctiform images, which are representative of static air bronchograms, or hyperechoic tubular images, which are representative of dynamic air bronchograms, corresponding to the complete loss of aeration. LUS was calculated as the sum of the points ranging from 0–36. Lung ultrasound was performed on days 1, 2, 3, 5, and 7 after patients were admitted to the ICU; these time points are called T1, T2, T3, T4, and T5, respectively. If the patient was intubated, the LUS scoring was performed before intubation within 24 h (T1) and on days 1, 2, 5, and 7 after intubation (T2, T3, T4, and T5, respectively).

### Statistical analysis

Statistical analyses were performed using STATA V12 (Stata Corp, College Station, TX, USA). All statistical tests were performed at an α risk of 5% (excluding interim analysis). Continuous variables are presented as the mean and standard deviation, subject to the normality of distribution (Shapiro-Wilk). In case of non-normality, these are presented as the median, quartiles, and extreme values. Qualitative variables are expressed as numbers and associated percentages. Graphic representations are associated with the analysis. Comparisons between groups were conducted systematically: (1) without adjustment, and (2) adjusted by regression model based on factors whose distribution could be unbalanced between the groups despite randomization.

RETRACTED

## Results

### Patient demographic characteristics

During the study period, 72 patients presented to the ICU in Wuhan with COVID-19 within one month; 43 patients were confirmed to be severe cases. Twenty-seven patients were excluded for the following reasons: five patients were intubated before transferring to our ICU, four patients died within 72 h, and 18 patients were not assessed by transthoracic lung ultrasound, and thus had no data. A total of 16 patients were included this study, of whom nine were intubated within 72 h after admission into the ICU, and seven patients were not intubated and treated with a non-rebreather mask, non-invasive ventilator (NIV), or high-flow nasal cannula oxygen therapy (HFNC). The demographics, clinical features, and outcomes of the sample are presented in Table 1. The mean participant age was 58.0 (47.0–68.0) years old, with a higher proportion of older patients in the intubated group than in the non-intubated group (P < 0.05). There were more male patients than female patients in both groups. Patient characteristics (BMI, SOFA, and PaO_2_/FiO_2_ value) were similar between the two groups (P > 0.05). The 28-day mortality rate of intubated patients was higher than that of non-intubated patients, and six patients in the intubated group and two patients in the non-intubated group died. Table 2 shows the evolution of respiratory parameters between the two groups on T1; no differences in respiratory rate, pulse rate, PH, PaCO_2_, PaO_2_/FiO_2,_ and SpO_2_ were found between the two groups.

**Table 1:** Patient characteristics at baseline, according to study group.

Parameter	All (n = 16)	Intubated group (n = 9)	Non-intubated group (n = 7)	P-value
Age (year)	58 (47–68)	68 (51–78)	54 (47–60)	<0.01
Gender (males/females)	9/7	6/3	3/4	0. 532
BMI	23.1 ± 4.3	22.4 ± 4.1	23.8 ± 4.5	0. 367
SOFA score	7.1 ± 2.8	6.1 ± 2.6	6.7 ± 2.7	0. 241
LUS 1st	11.3 ±4.6	10.6 ± 4.9	12.1 ± 4.2	0. 25
PaO_2_/FiO_2_	146 (134–168)	144 (132–167)	148 (136–168)	0.781
HFNC	5	3	2	
NIV	4	2	2	
28-day mortality (%)	8 (50%)	6 (66.7%)	2 (28.5%)	<0.01

Data are presented as the number of patients, mean ± SD, or median and interquartile interval (25 to 75%).

RETRACTED

**Table 2:** Evolution of respiratory parameters between the two groups on T1.

Variables	Intubated group (n = 9)	Non-intubated group (n = 7)	P-value
Respiratory rate, breaths/min	26 ± 5	28 ± 4	0.21
Pulse rate, beats/min	106 ± 17	103 ± 19	0.91
PH value	7.32 ± 0.23	7.35 ± 0.19	0.78
PaCO_2_, mmHg	41.4 ± 7.8	45.2 ± 12.1	0.39
PaO_2_/FiO_2_	140.1 ± 7.7	137.8 ± 5.9	0.75
SPO_2_	94.2 ±3.1	95.1 ± 4.2	0.68

Data are presented as number of patients, mean ± SD, or median and interquartile interval (25 to 75%).

### Comparison of LUS between the two study groups

Fig 1 shows the changes in LUS within seven days of ICU admission for non-intubated patients (n = 7). The average LUS was 10.7 ± 1.4 on T1 and 10.3 ± 2.9 on T5, and the lowest LUS was 10.7 ± 1.1 on T3. There was no significant difference in LUS among time points. Fig 2 shows the changes in LUS of intubated patients (n = 9) at different time points. The LUS within 24 h before intubation was 12.8 ± 1.3. LUS was significantly higher at T5 than T1 (P < 0.05), but the scores did not significantly differ from T1 to T4. Fig 3 shows that the LUS of intubated patients, 12.8 ± 1.3, was significantly higher than the LUS of the non-intubated patients at T1, 10.7 ± 1.4 (P < 0.05). Fig 4 shows a comparison of the oxygenation index of the two groups of patients: 140.1 ± 7.7 *vs*. 137.8 ± 5.9 on T1. There was no significant differences in oxygenation index between the two groups.

**Fig 1:** Lung ultrasound score of non-intubated patients (n = 7) within 7 days.

**Fig 2:** Lung ultrasound score of intubated patients (n = 9) within 7 days.

**Fig 3:** Comparison of lung ultrasound score in the two study groups on T1 (*P* = 0.05).

**Fig 4:** Comparison of oxygenation index in the two study groups on T1.

## Discussion

The high contagiousness of SARSCoV-2 and the risk of transporting unstable patients with hypoxemia and hemodynamic failure make chest CT a limited option for patients with suspected or established COVID-19. Lung ultrasonography generates results that are similar to those of chest CT and superior to standard chest radiography when evaluating pneumonia and/or adult respiratory distress syndrome (ARDS), with the added advantages of ease of use at point of care, repeatability, absence of radiation exposure, and low cost [13].

The most important clinical manifestations of respiratory failure in patients with COVID-19 are hypoxemia and increased work of breathing. Attention should be paid to the different effects of different oxygen therapy concentrations to avoid prolonged high-concentration oxygen therapy [14]. During the treatment process, deciding when to switch from non-invasive ventilation or high-flow oxygen therapy to invasive mechanical ventilation and how to dynamically assess lung condition changes can be challenging. For critically ill patients with COVID-19, the difficulty of accurately assessing lung conditions is greatly increased due to the inability of doctors to use stethoscopes in protective clothing, as well as due to the use of lung CT to repeatedly evaluate patients' lung conditions in special circumstances. Several studies on non-COVID-19 patients have demonstrated that lung ultrasound is accurate for assessing positive end-expiratory pressure, prone position-induced lung recruitment, lung reaeration following antimicrobial therapy in ventilator-associated and community-acquired pneumonia, and lung reaeration associated with the resolution of various forms of pulmonary edema [8–10]. Soummer et al. first proposed and successfully applied this method to assess the changes in lung ventilation for patients after offline extubation, and they confirmed that patients with LUS > 14 had a significant increase in intubation rate after offline extubation [15]. An experienced sonographer can perform this examination within five min, and brief training and about 25 supervised exams seem to be sufficient to achieve a basic ability to perform the task [16]. A prior study showed LUS’s ability to influence clinical decisions in up to 50% of ICU patients [17].

RETRACTED

In this study, the LUS of the intubated group on T1 (within 24 h before intubation) was higher than that of the non-intubated group. However, oxygenation index and respiratory rate, the conventional indicators to decide whether to intubate critical care patients, did not significantly differ between the two groups at the same time point. The obvious difference indicates that the LUS may be a more accurate indicator of ideal intubation timing than the oxygenation index and respiratory rate. LUS could dynamically assess the ventilation status of the two patient groups during treatment, and provided earlier prediction of pulmonary ventilation status and disease deterioration. An LUS = 12 may be a warning for intubation or exacerbations in critically ill COVID-19 patients. Clinicians need to closely observe the patient’s condition and consider the possibility of tracheal intubation according to the patient's situation.

A unique syndrome of hypoxic COVID-19 patients has been described (labelled “the happy hypoxic”) who are mentally alert and lack significant respiratory distress despite hypoxia that would usually prompt treatment, sometimes with profoundly low oxygen saturations [18]. According to our experience in treating patients with severe COVID-19 in Wuhan, most patients are more tolerant to hypoxia, and patients with a low oxygenation index often have no obvious symptoms of chest tightness, shortness of breath, or mild symptoms, which are inconsistent with clinical indicators. There is no evidence that choosing early intubation instead of NIV or HFNC improves outcome: early reports suggest intubated patients remain on ventilators for extended periods and mortality rates appear high. A retrospective cohort study of 191 patients in Wuhan showed that mortality rate was significantly increased after intubation; 57% of patients died after mechanical ventilation treatment, and patients often had complications such as septic shock, ventilator-associated pneumonia (VAP), and deep vein thrombosis after intubation [19]. Intubated patients are thought to pose a lower risk of viral dispersion to staff. However, both the process of intubating and extubating are high risk to staff, and there are reports of accidental ventilator circuit disconnection when intubated. Therefore, judging the timing of intubation and mechanical ventilation treatment is a concern for doctors in the emergency department and ICU, but no recent study has found the best clinical indicators for evaluation. Lung ultrasound is an ideal inspection method in addition to the gold standard CT examination, and may be one of the most effective tools for judging intubation time. According to our experience, the accuracy of bedside ultrasound in evaluating severe and critical COVID-19 patients is significantly better than its accuracy in evaluating mild patients. The reason may be that the exudation of mild COVID-19 patients is often not obvious, and the lesions are deep and/or pleural, and not accumulated. Lung ultrasound’s usefulness is limited, especially in cases of early or mild COVID-19. According to previous studies, LUS is a semi-quantitative assessment of lung ventilation by ultrasound. An LUS of 14 (scored out of 36) may thus be an indicator for intubation in patients with respiratory failure. In this study, the LUS before intubation was 12.8 ± 1.3, which is lower than the score suggested by the previous study (14 points). The reason for this may be that the primary CT manifestation of the patients in the group was pulmonary exudation without obvious consolidation or atelectasis, which accounts for 3 points in the LUS. Because the behavior of ARDS caused by COVID-19 differs from that caused by other diseases, the patient's LUS for COVID-19 shows mainly a large number of B lines in both lungs, and is lower than normal ARDS patients, which show consolidation in some parts of the lung. Most patients with mechanical ventilation have secondary bacterial infections or poor sputum drainage, which may cause some consolidation of the lungs and atelectasis, leading to a significant increase in LUS after intubation [20–22].

RETRACTED

## Conclusions

This study indicates that LUS may be an effective tool for assessing the timing of intubation in patients with SARS-CoV-2 pneumonia/ARDS. The intubation of critically ill patients with COVID-19 is mostly due to respiratory failure, but there is also a small number of patients who undergo intubation due to secondary acute heart failure or airway obstruction [23]. Thus, an ultrasound may be employed to evaluate cardiac function and other conditions as part of a comprehensive COVID-19 assessment. As this study is a retrospective study, the number of patients included in this investigation is relatively small, and further large-scale prospective studies are needed to confirm our findings.

## Supporting information

S1 Data (XLSX)
